# The Progress of Functional Magnetic Resonance Imaging in Patients with Poststroke Aphasia

**DOI:** 10.1155/2022/3270534

**Published:** 2022-04-21

**Authors:** Jinping Tang, Xuli Xiang, Xianglin Cheng

**Affiliations:** ^1^The First Affiliated Hospital of Yangtze University, Jingzhou 434000, Hubei, China; ^2^The Second People's Hospital of Gongan County, Jingzhou 434000, Hubei, China

## Abstract

Aphasia after stroke is one of the common complications of cerebral infarction. Early diagnosis and treatment of aphasia after stroke is of great significance for the recovery of language function. At present, there are different views on the pathogenesis of aphasia after stroke. Functional magnetic resonance imaging (fMRI) can reflect the brain function, brain tissue metabolism, and the level of brain local blood flow. It has the advantages of noninvasive, high resolution and sensitivity, low price, and so on. It has been widely used in the study of sensory aphasia after stroke. This study focuses on the development of functional magnetic resonance imaging in patients with poststroke aphasia and summarizes the published studies on functional magnetic resonance imaging in patients with poststroke aphasia. *Evidence acquisition*: A literature search was conducted in PubMed, Hindawi, PLoS, IEEE, Wiley, ScienceDirect, Springer, EMBASE, and web of science, with the keywords of “stroke” and “Aphasia” and “functional magnetic resonance imaging”, “RS fMRI”, or “DTI”, to review the research of functional magnetic resonance imaging in patients with aphasia after stroke. The results included clinical evaluation, diagnostic scale, and imaging analysis; the study design was a randomized controlled trial, case series and case report, and observational study. A total of 67 articles were identified in the first search and 43 after the second search. Based on the analysis of 43 selected articles, 19 articles were included, and 24 articles were excluded. The selected information is shown in Table 1. Eleven of them did not contain imaging-related data. Six articles are related review articles. Four studies were conducted on patients without poststroke aphasia. Three studies studied the effect of poststroke aphasia on patients' social participation.

## 1. Introduction

Stroke is caused by cerebral circulation and blood circulation disorder, which causes cerebral tissue ischemia and hypoxia to cause softening and necrosis. Incidence rate, disability rate, and mortality rate are all higher than the study of [1]. With the gradual increase of the aging trend of the population in China, the incidence rate of stroke increases gradually. Cerebral infarction is the most common stroke type, accounting for 69.6% to 70.8% [2] of stroke in China. Aphasia is a common symptom of cerebral infarction, accounting for 21% ∼ 38% of patients with acute cerebral infarction. Language disorders seriously endanger the physical and mental health of patients, bring mental and economic pressure to patients and families, and increase social burden [3, 4]. Many patients have aphasia. Aphasia refers to acquired language dysfunction, that is, the acquired language ability. Due to the language processing disorder caused by the brain damage of language function, the ability to understand and form language is impaired [5]. Aphasia patients can have various language or speech disorders, most of which are limited or even lost in spontaneous language, naming, retelling, reading, writing, and understanding. Aphasia seriously affects the daily communication ability of patients. Language is an indispensable part of cognitive function. At the same time, it also affects the memory, understanding, and other functions of patients [6, 7]. Moreover, the occurrence of aphasia seriously affects the quality of life of stroke patients and their ability to return to family and society and causes a heavy burden on patients, family, and society. Aphasia after stroke is caused by direct damage to the cerebral cortex or the brain-related network dysfunction after stroke, and the incidence rate is about 30% [8,9] of stroke patients. Early diagnosis and treatment of aphasia after stroke is of great significance for the recovery of language function, Table 1.

In recent years, functional magnetic resonance has made some achievements in the diagnosis and treatment of poststroke aphasia. Functional brain imaging, such as functional magnetic resonance imaging (fMRI), is a popular method to study aphasia. FMRI mainly includes diffusion tensor imaging (DTI) and blood-oxygen-level-dependent (BOLD) imaging. DTI is the only new magnetic resonance imaging technology developed rapidly in recent years, which can image the structure of brain white matter in vivo. It provides the possibility to study brain white matter fibers and makes up for the shortcomings of other neuroimaging technologies in this regard. It uses the diffusion anisotropy of water molecules in biological tissue to image the biological tissue structure, which can provide white matter fiber information that other neuroimaging technologies cannot provide and can visualize the white matter fiber neural pathway in 3D. Therefore, DTI has become one of the most popular fMRI techniques in brain function research and clinical application. Resting-state functional MRI (rs-fMRI) belongs to BOLD fMRI. Because the detection of rs-fMRI does not require the patient to perform specific language tasks, it is simple and easy, and the patient's compliance is good. It has developed rapidly in recent years. It has become the most commonly used tool for the study of language function recovery after stroke and is widely used in the study of neurological diseases and mental disorders.

However, there is no research on the application of RS fMRI and DTI in poststroke aphasia. Therefore, this paper reviews the research progress of functional magnetic resonance imaging in patients with poststroke aphasia to provide an overall outline of the impact of fMRI in poststroke aphasia.

## 2. Poststroke Aphasia

Modern studies generally believe that poststroke aphasia is a clinical syndrome of patients with abstract signal thinking disorder caused by central neuropathy and then loss of the ability of oral and written expression and comprehension. It is an acquired language disorder caused by the damage of language distribution network with extensive language distribution in the cortex and subcortical structure of language dominant hemisphere [10]. Aphasia can be caused by many diseases, especially stroke. The pathogenesis of aphasia caused by stroke is mostly caused by the damage of brain language functional areas and related nerve fibers. Due to the obstacles in language expression, understanding and related reading and writing skills, the social ability of stroke patients with aphasia is affected, which prevents them from returning to society [11, 12].

Aphasia is the loss or damage of language function caused by brain damage. It is common in cerebrovascular diseases, brain trauma, brain tumors, brain inflammation, and so on. Most of the patients are caused by acute cerebrovascular disease in the left (dominant hemisphere). Aphasia patients often show different degrees of defects in oral expression, listening comprehension, retelling, naming, reading, and writing [13]. Clinically, aphasia is divided into Broca aphasia, Wernicke aphasia, conductive aphasia, transcortical motor aphasia, transcortical sensory aphasia, mixed transcortical aphasia, naming aphasia, and complete aphasia according to the characteristics of patients' language disorders [14, 15].

The pathogenesis of traditional aphasia includes localization theory and antilocalization theory. Aphasia localization theory refers to the theory that language activities are related to specific parts of cerebral cortex, such as Broca and Wernicke cortical language areas (Geschwind-Wernicke language model theory). Language information is introduced into Wernicke area and processed and transmitted to Broca area by arcuate fiber bundle. Finally, Broca area processes the information and transforms it into language activities [16]. Most scholars believe that speech disorders caused by lesions in different parts of the left cerebral hemisphere have their own characteristics, including Broca aphasia caused by damage to the Broca area in the posterior part of the left inferior frontal gyrus, Wernicke aphasia caused by damage to the Wernicke area in the posterior part of the temporal transverse gyrus of the auditory cortex, conductive aphasia caused by damage to the projection fibers or arcuate bundles between the temporal-parietal and frontal lobes, and complete aphasia caused by Broca area, Wernicke area, basal ganglia area, and insula damage [17–19]. However, localization theory cannot well explain aphasia caused by subcortical structures, such as white matter or nuclear lesions. The other is the antipositioning theory, which holds that language activities are formed by the participation of the whole brain; that is, the occurrence of language dysfunction is not caused by the damage or loss of function of specific brain regions but involves the dysfunction of the whole brain neural network [20]. In addition, the more typical language neurobiology model is the dual flow structure model similar to the visual system proposed by Ungerleider and Haxby in 1994. This model proposes a method to map auditory speech to the dorsal flow of pronunciation (movement) and auditory speech to the ventral flow of semantics; that is, backflow mainly supports speech generation and speech perception, while the abdominal flow is responsible for semantic understanding/processing, which may be more in line with the mechanism of language network generation and understanding. At present, the classification of aphasia is mainly divided into Broca, Wernicke, conductive, transcortical (motor and sensory), complete, nominal aphasia, and some rare types of aphasia [21]. Understanding the mechanism and classification of aphasia is helpful to further explore the changes in brain function in patients with poststroke aphasia after treatment. At present, functional magnetic resonance imaging is gradually more and more widely used in the field of poststroke aphasia.

## 3. Principle and Background of Functional Magnetic Resonance Imaging

Functional magnetic resonance imaging (fMRI) mainly includes diffusion tensor imaging (DTI) and blood-oxygen-level-dependent (BOLD) imaging. BOLD fMRI is an MR imaging technology that uses the change of T2-weighted image of local tissue caused by the change of the ratio of oxygenated hemoglobin to deoxyhemoglobin in the local blood of brain activity area, so that the local activity function of brain tissue can be reflected on T2-weighted image, which can not only reflect the patient's brain function, brain tissue metabolism, and the level of brain local blood flow (Figure 1). Moreover, it has been widely used in the study of sensory aphasia after stroke because of its noninvasive, high resolution, sensitivity, and low price [22]. BOLD fMRI is mainly divided into task fMRI and resting fMRI. During the implementation of task fMRI, patients need to perform specific tasks or receive preset external stimuli to induce neuronal activities in different states of the brain, so as to obtain the activation map of the difference in brain neuronal activity signals and to reveal the law of brain activity in specific task states [23]. Resting state functional MRI (RS fMRI) and diffusion tensor imaging (DTI) overcome some defects of task fMRI. The detection of RS fMRI or DTI does not require the patient to perform specific language tasks. It is simple and easy, and the patient's compliance is good. It has developed rapidly in recent years. It has become the most commonly used tool for the study of language function recovery after stroke and is widely used in the study of neurological diseases and mental disorders [24].

## 4. Research Progress of rs-fMRI

Rs-fMRI reflects a long-range coherent functional model and is the spontaneous activity of the central nervous system in the basic state. At present, the research on resting brain network has two directions: one is seed-based correlation analysis (seed-based correlation analysis) and independent component analysis (ICA), which studies the synchronization of time series in distant brain regions and the functional connection between brain regions [17, 25]. The second is the analysis method of regional consistency (ReHo) and amplitude of low-frequency oscillation (ALFF) to study the synchronization of local brain regions in time series and the degree of spontaneous neural activity in local brain regions [8, 26]. Brain functional connectivity analysis is a common processing method of rs-fMRI.

According to traditional linguistics, Broca area is mainly responsible for language generation, Wernicke area (posterior part of left superior temporal gyrus) is responsible for language acceptance and understanding, and the arcuate bundle between Wernicke area and Broca area is responsible for the traffic connection between them [27]. Krishnamurthy S. [28] found that there is a language understanding network centered on the posterior temporal gyrus of the dominant hemisphere in the resting state, which may be the neural basis of the brain's language understanding function. Yi K. [29] found that the recovery of language function is accompanied by the dynamic change of functional connection: the functional connection coefficient of language neural network in stroke patients in the acute stage is significantly reduced, and the functional connection coefficient of language neural network in chronic stage is enhanced. It was also found that high-risk patients had reduced resting functional connectivity. Naeser M. A. [30] studied 13 patients with poststroke motor aphasia with left hemisphere injury. It was found that the average functional connectivity index of the left frontal-parietal lobe decreased, accompanied by an obvious loss of language understanding. With the improvement of language comprehension, the average connectivity index of the left frontoparietal lobe also increased. Therefore, Naeser Ma [30] believes that brain tissue injury may affect language understanding ability by changing the functional connection of brain interval, and the recovery of language function is also related to the change of functional connection.

Brain functional connectivity analysis was used to observe the effect of intervention measures on brain functional connectivity. Patients with motor aphasia after stroke can recover spontaneously without intervention. The recovery is obvious in the acute phase and slows in the chronic phase [31]. However, studies have shown that the recovery effect of language rehabilitation treatment in the acute stage of motor aphasia after stroke is almost twice that of natural recovery [32]. Lee J. K. [33] used resting-state functional connectivity to evaluate the effect of naming in the treatment of poststroke motor aphasia. Eight patients with poststroke motor aphasia received 12 treatment courses of improved naming. Before treatment, the activation of the right middle temporal gyrus gradually shifted to the left with the improvement of language function.

## 5. Research Progress of DTI

DTI is a new image expression method based on conventional magnetic resonance imaging technology. DTI is a special form of MRI, which can not only display the signal intensity of each voxel but also calculate the specific data of tensor direction in three-dimensional space [34]. Then, the single arrow displayed by each voxel is sorted according to the difference in nerve bundle direction to generate a group of direction arrows. Then, the direction arrows of each group are processed through the processing of image data to form a linear image of the nerve bundle. DTI allows us to objectively study poststroke aphasia from the perspective of the structural connection of white matter fibers. Zavanone C. [35] believes that DTI can be used as a good indicator of peripheral nerve regeneration and a noninvasive diagnostic tool for a variety of nervous system diseases. Carragher M. [36] and other researchers collected aphasia patients with different severity and examined the damage of white matter fiber bundle with DTI. They found that DTI examination was helpful to predict the severity of language disorder in aphasia patients after stroke. At present, the research related to DTI mainly involves the occurrence mechanism, recovery mechanism, and prognosis of aphasia.

The formation mechanism of poststroke aphasia has been unclear. At present, it is recognized that the occurrence of aphasia is related to the damage of language functional areas of the cerebral cortex. The lesion location of poststroke aphasia is closely related to the specific functional language area and arcuate fiber bundle of the brain. The injury of arcuate fiber bundles in specific functional language areas of the brain is the main factor leading to aphasia after stroke, which can also be used as an imaging auxiliary tool to evaluate the patient's condition [37]. François C. [38] found that patients with Broca aphasia, Wernicke aphasia, and conductive aphasia had different degrees of damage to the arcuate fiber bundle, and the damage location was related to the type of aphasia: Patients with Broca aphasia mainly had damage and displacement of the integrity of the front end of the arcuate fiber bundle, and patients with Wernicke aphasia mainly had middle and rear damage. In patients with conductive aphasia, the central part of the arcuate fiber bundle on the functional side was mainly damaged. Zhang J performed DTI and fiber bundle imaging on patients with language disorders to check the integrity of the arcuate bundle. DTI and fiber bundle imaging showed that the arcuate bundle was seriously damaged [39]. Patients with sports aphasia have left arcuate fasciculus injury with anterior changes in varying degrees, and the degree of injury is positively correlated with the severity of aphasia, indicating that arcuate fasciculus is an important channel for the communication between anterior and posterior language function zoning. Yao J and others believe that arcuate fiber bundle damage and lesions in cortical language functional areas such as Broca area and Wernicke area can cause conductive aphasia. If the lesion is close to the Broca area, the patient's language disorder is similar to Broca aphasia; if the lesion is close to the Wernicke area, it is similar to Wernicke aphasia [40]. It can be seen that the research on the mechanism of aphasia using DTI breaks the previous understanding of the mechanism of aphasia. For example, the Broca area of Broca aphasia patients is not necessarily damaged, and conductive aphasia can also be caused by lesions in cortical language functional areas such as the Broca area and Wernicke area. These findings make the mechanism of aphasia more complex and need more in-depth research.

The application of DTI makes us to have a deeper understanding of the rehabilitation mechanism of aphasia after stroke. Brain plasticity and language function reorganization are generally accepted at present. Some scholars believe that the study of arcuate fiber bundle by DTI shows that the study of brain white matter fibers can explore the recovery mechanism of aphasia from the level of brain structural changes to a certain extent [41]. Gleichgerrcht E. [42] included 6 patients with left hemisphere stroke with moderate and severe nonfluent aphasia. DTI was tested before and after 75 times of intensive speech therapy. It was found that the number of arcuate fiber bundle fibers and the volume of arcuate fiber bundle were significantly increased after treatment compared with that before treatment, suggesting that the recovery of speech function was related to arcuate fiber bundle remodeling. After one month of intensive rehabilitation treatment, Forkel S. J. found that the number and integrity of left arcuate fiber bundles in a patient with poststroke aphasia also increased [43]. These studies show that the arcuate fiber bundle of patients with poststroke aphasia will change structurally after speech intervention. Detecting this change by DTI will help to explore the recovery mechanism of aphasia.

The prognosis of aphasia after stroke is of great concern to clinical workers and patients. The prognosis prediction of aphasia patients after stroke has very important guiding significance for the formulation of the rehabilitation treatment plan and rehabilitation duration. The lesion location of the arcuate fiber bundle can predict speech rate, information content, overall efficiency, and naming ability [44]. Keser Z. believes that arcuate fiber bundle lesion load (lesion size and location) can predict speech fluency and naming ability in patients with poststroke aphasia [45]. Sanches C. [46] used DTI to study the recovery and prognosis of aphasia. It shows that the arcuate fiber bundle has clinical value in predicting the prognosis of aphasia after stroke.

In conclusion, DTI has irreplaceable advantages over other neuroimaging methods in the study of the white matter fiber pathway. At present, the research on poststroke aphasia using DTI has been preliminarily carried out, involving the discussion of the occurrence and recovery mechanism of aphasia and the prediction of prognosis, and also reflects its certain clinical application value. However, there is still a lack of research on the characteristics and differences of lesion location and mechanism between different types of aphasia, which needs more in-depth or detailed research. As an important pathway of brain nerve signal transmission, the cerebral white matter fiber bundle plays an important role in the occurrence of poststroke aphasia, but its mechanism has not been clarified. DTI technology can be used for in-depth research to objectively and effectively evaluate poststroke aphasia, explore the rehabilitation mechanism of poststroke aphasia, and predict the prognosis of poststroke aphasia patients.

## 6. Conclusion

The mechanism of language disorder in patients with poststroke aphasia has not been fully explained. At the time of acute cerebral infarction, there is low perfusion and low metabolism in the infarct area, and the place where the metabolic rate decreases the lowest is in the ischemic infarct area. At the same time, it is also found that the metabolic rate decreases in the ipsilateral language functional area; that is, the low metabolism in the language functional area may be the pathogenesis of aphasia [47]. This suggests that we can properly restore the perfusion and metabolism of the language center in the rehabilitation treatment of aphasia, so as to improve the language function. Functional magnetic resonance imaging technology provides a favorable clue to explore the pathogenesis and recovery mechanism of aphasia after stroke and provides a theoretical basis for the rehabilitation treatment of the brain. Rs-fMRI to evaluate the changes of language network functional connectivity in patients with poststroke motor aphasia is not only of great value for the discussion of aphasia occurrence and rehabilitation mechanism but also has a good application prospect for the early diagnosis, rehabilitation prognosis, and curative effect evaluation of poststroke motor aphasia. However, the current research results are quite different, and the potential recovery mechanism of motor aphasia after stroke has not been fully clarified. Rs-fMRI processing method still faces many major challenges. As an important pathway of brain nerve signal transmission, the cerebral white matter fiber bundle plays an important role in the occurrence of poststroke aphasia, but its mechanism has not been clarified. DTI technology can be used for in-depth research to objectively and effectively evaluate poststroke aphasia and explore the rehabilitation mechanism of poststroke aphasia. However, there is still much room for improvement in the study of functional magnetic resonance imaging in poststroke aphasia. With the development of imaging technology, functional magnetic resonance imaging may play a more important role in the individualized treatment evaluation of patients with poststroke aphasia in the future.

## Figures and Tables

**Figure 1:** FMRI working principle.

**Table 1:** Literature inclusion.

Authors	Study design	Authors	Study design
Gray M.	Case report	François C.	Retrospective study
Lee J. K.	RCT	Zhang J.	Retrospective study
Inatomi Y.	Case report	Fridrikson J.	RCT
Stampacchia S.	RCT	Yin J.	Case report
Allendorfer J. B.	Case report	Yi K.	Case report
Wang Y.	Retrospective study	Kawano T.	Retrospective study
Dickens J. V.	Retrospective study	Iorga M.	Retrospective study
Kristinsson S.	RCT	Ellis C.	Retrospective study
Kim G.	Retrospective study	Krishnamurthy S.	Case report
Hybinette H.	Retrospective study	Brady MC	RCT

RCT: randomized controlled trial.

## Data Availability

The datasets used and analyzed during the current study are available from the corresponding author upon reasonable request.
